The article "Analysis on the Nonlinear Impact of Financial Risks on CO2 Emissions: Designing a Sustainable Development Goal Framework for Asian Economies" was published in 2022. Journal: J Environ Public Health.

# Analysis on the Nonlinear Impact of Financial Risks on CO_2_ Emissions: Designing a Sustainable Development Goal Framework for Asian Economies

**DOI:** 10.1155/2022/8458122

**Published:** 2022-08-30

**Authors:** Xuan Huang, Meihua Chen

**Affiliations:** ^1^School of Software and Internet of Things Engineering, Jiangxi University of Finance and Economics, Nanchang, Jiangxi 330013, China; ^2^School of Public Administration, Nanchang University, Nanchang, Jiangxi 330031, China

## Abstract

For the purpose of coping with or eliminating the influence of carbon dioxide emissions effectively, it is crucial to apply the green investment models to carry out a qualitative analysis of carbon dioxide emission evolution. The effect of financial risks on the implementation of the carbon dioxide emission limit is essential for the distribution of resources, and it is necessary to summarize the patterns and make innovations in the process of limiting the emissions of carbon dioxide effectively. In the case of fully complying with the principles of low-carbon economic development and related policy protection, the appropriate model for low-carbon economic development is identified. In this article, the multivariate primary nonlinear model is applied to the analysis of the nonlinear influence of financial risks on carbon dioxide emissions to cope with the problem of financial risks on carbon dioxide emissions at present. In this method, a multivariate primary nonlinear model is established based on the detailed analysis of the financial development features, and the parameters are optimized mainly from various aspects such as the structure of the model, the features of data, and the dynamic changes of the model so as to obtain the optimal values for the parameters of the constructed multivariate primary nonlinear model. The results of the practical case analysis indicate that the influence of financial risks on the limits of domestic carbon dioxide emissions is differentiated in accordance with the results and related categories. Only in this way can the regional division of carbon emission factors be properly classified. The relationship between economic growth and carbon emission increase and changes indicates that effective strategies for carbon emission reduction should be adopted. The established panel data model is used to carry out an in-depth analysis of the influence of carbon dioxide limitations in Asian countries.

## 1. Introduction

The implementation of real-time, rational, and accurate monitoring of carbon dioxide emissions can also provide a theoretical basis for the analysis of the decisions made by the relevant authorities for environmental protection inspection, which is of important significance for the increasing number of financial risk projects that are springing up. A detailed analysis of the financial risks is carried out to explore the issues and defects of the carbon dioxide emission process so as to develop more scientific and effective training and upgrading programs in the later stage. In the process of analyzing the evolution of traditional carbon dioxide emissions, carbon dioxide emissions and real-time risk alerts are also effective processes for data acquisition and analysis processes with regard to carbon dioxide emission equipment [1–3]. The relevant index data are collected from the carbon dioxide emission process, and the corresponding feedback is given. The data obtained are used to analyze the performance of carbon dioxide emissions, analyze the operational status of carbon dioxide emissions, diagnose the causes of faults, and monitor the root causes of the faults. Carbon dioxide emissions and real-time risk alerts are an integral part of carbon dioxide emission management and system integration, which has provided specific data for the operation and maintenance of carbon dioxide emissions. With regard to the development of financial risk, green investment, and carbon emission, they have attracted more and more attention from research scholars, and it has been proved by facts that there is a huge gap in the changes of carbon emissions under different systems in various environments. There is a direct link between economic development at its highest speed and carbon emissions under tremendous financial risks. The countries in Asia have already made their commitment to climate development, mandatory development of a low-carbon lifestyle, and the truly effective improvement via the pathway of carbon reduction, which has determined the qualitative change in the living environment and shouldered the corresponding social responsibilities. At the same time, the structure of the industry is being overhauled and developed, which, however, is a long process of development [4–6]. The relationship between the economic growth and the carbon dioxide emissions in the country has a relatively prominent gap among various regions, and some information indicates that in accordance with the total carbon emissions calculated, a manual distinction is made between regions to carry out the related studies based on the factors in different regions. For the purpose of effectively coping with the problem of environmental pollution, Asian countries have coordinated their economic development with environmental protection and given full play to the advantages of their respective environmental resources [7, 8]. With regard to the increasing financial risks, it requires that the emerging Asian countries in Asia should focus on the development of the environment and the economy in harmony with the production processes to improve production efficiency and make full use of the limited resources so as to better boost the economic development of the countries in Asia and seize the opportunity in the financial risk prevention process. However, due to the demand for the investment of a large amount of capital and labor costs under the financial risks in the countries, it can lead to a decline in the economic growth of Asian countries; that is, the high cost of economic development will influence the environment and the continuous development of the economy, which will have a negative effect on the sustained development of Asian countries; with regard to the competitors, it is necessary to spend additional costs. Where the evidence indicates that the economic entities of Asian countries reach a certain level, environmental sustainability will present growth at a doubled speed. All the regions that exceed this level are distributed in the eastern part, followed by the central region, and those at the lowest level are located in the western part. With the continuous progress of the green economy development in Asian countries, the relatively large-scale green economies in Asian countries have been developed rapidly, and more green economy sustainability projects have emerged. The green economy sustainability development is analyzed in detail to explore the issues and defects of the green economy development process so that more scientific and effective training programs and upgrading plans can be developed in the later stage. At present, with the demand for the green economy sustainable development, it is required that the Asian countries with the green economy sustainable development should be able to implement a one-stop service system that can offer strong support for life and achieve the highest economic benefits for the sustainable growth of the whole green economy, which is the overall goal of Asia countries in pursuit of green economy sustainability [9, 10].

With the continuous advancement of Internet technology and the increasing technological level, different financial developments based on the Internet have started to emerge. However, how to acquire the specific content sources from the initial financial development data that lack financial content definition and specific description has become a huge challenge for the multivariate primary nonlinear operation of financial growth at present. Since the financial development signal falls into a type of time sorting, it is feasible to apply the multivariate primary nonlinear model based on its concealed features. So far, the other classification methods are relatively homogeneous and inaccurate in obtaining the features of financial growth. The multivariate primary nonlinear model is applied to the process of nonlinear effect analysis of carbon dioxide emissions. This method allows for the use of financial development as current prior knowledge in the process of carbon dioxide emission nonlinear effect analysis in accordance with the spatial features of financial growth. The information gain method is extracting the features from the financial development content. Constrained spatial weights for multivariate primary nonlinear models for integration with spaces of high similarity on the basis of acquired financial information, respectively, are to build multivariate primary nonlinear operational models of financial development. Through the construction of the multivariate primary nonlinear model system, it can be observed that the model parallelization has substantially improved the efficiency and timeliness. The multivariate primary nonlinear model is introduced into the autonomous multivariate primary nonlinear operation of financial growth, which can implement accurate and fast multivariate primary nonlinear operation accordingly [11, 12]. At the same time, in combination with the rhythmic features of financial development, the accuracy of the multivariate primary nonlinear operation for financial growth based on the RFAM model can be improved to 67.9%. The visual analysis of the multivariate primary nonlinear operation of financial growth is implemented on the basis of the multivariate primary nonlinear model. In the implementation stage, the maximum reduction of carbon dioxide emissions is required. The general environment in the Asian countries studied has entered a new course, and the differences brought about by the various economic growth and economic situations of each region have a decisive effect on the local carbon emissions, changes, and roles. It is necessary to make the green investment that produces lower carbon emissions, ensures greener growth, and results in less energy loss. Due to the relatively huge differences in economic growth within a region, the development of reasonable and scientific policy standards for carbon emission reduction in accordance with the level of economic growth and the status of carbon dioxide emissions in the region of each country as the practical case may become a preferred path to develop a low-carbon economy in the country. With regard to countries in the development of low-carbon emission reduction policies, it is necessary to consider the details in different regions, different areas, as well as the corresponding urban basic resources, environmental pollution status quo, and industrial structure features; consider the basic situation of the respective economic development, social situation, energy availability, and green-related policies in each country effectively; proactively identify domestic demand; explore the suitable models for their own regional carbon dioxide emissions and renewable energy quotas; and guide the entire society to make concert effort in saving energy and improving energy efficiency so as to reduce the pollution of the environment [13, 14].

Studies have shown that there are obvious gaps in the relationship between economic growth and carbon dioxide emissions in Asian countries. Some data show that after calculating the total carbon emissions, the regions are divided manually, and the factors of different regions are studied. Questions are raised about the arrangement of such pre-distinguished regions. It should be based on regional carbon emissions and economic disturbances, regular distinctions are made, and then distinctions are made according to results and categories so that regional divisions and research on carbon emission factors can be implemented, study the relationship between economic growth and carbon emission growth, and suggest the effective implementation of carbon reduction strategies.

## 2. Construction of a Measurement Model for the Impact of Financial Risks on GHG Emissions in Asia

This article mainly focuses on the relationship between economic finance and the growth of environmental carbon emissions. With regard to the stochastic multivariate primary nonlinear model, it can be established based on the most serial time series and applied in the process of analyzing the nonlinear effect of financial risks on carbon dioxide emissions on a large scale. There are *N* states that exist in the model. It is assumed that the *N* states are *S*={*S*_1_, *S*_2_,…, *S*_*n*_}, then the state at the moment *t* can be denoted by *q*_*t*_. The transfer matrix between the different states is represented by *A*={*a*_*ij*_}. Thus, the following expression can be obtained:

(1) $$\begin{array}{c} \alpha_{ij}\left(k\right)=P\left[q_{t+1}=S_{j}|q_{t}=S_{i}\right],\;1\leq i,j\leq N. \end{array}$$

With regard to any state in a transfer, the other states can be reached; while in some other RFAM, only certain transfers between states can occur, that is, *a*_*ij*_ > 0 is established for some *i*,*j* only. For each state, the external value is available for only one observation; the observation vector obtained is correlated with the state of the system, and this relationship can be discrete or continuously distributed.

However, for the observation with a continuous distribution, the distribution of the corresponding observation vector probability in the state *j* can be expressed as the following:

(2) $$\begin{array}{c} b_{j}\left(v_{t}\right)=P\left[v_{t}|q_{t}=S_{j}\right],\;1\leq j\leq N. \end{array}$$

In general, the distribution of probability is taken as a mixed Gaussian distribution, that is, the following can be obtained:

(3) $$\begin{array}{c} b_{j}\left(v_{t}\right)=\sum_{m=1}^{M}\omega_{j,m}N\left(o_{t},\mu_{j,m},\Sigma_{j,m}\right), \end{array}$$

where *M* stands for the number of mixed Gaussian distributions, *ω*_*m*_ stands for the positive mixed weights, and *N*(*o*_*t*_, *μ*_*j*,*m*_, Σ_*j*_, *m*) represents the situation of the *n*-dimensional Gaussian distribution.

(4) $$\begin{array}{c} \pi_{i}=P\left[q_{1}=S_{i}\right],\;1\leq i\leq N, \end{array}$$

Hence, RFAM can be summarized as three groups *λ*=(*A*, *B*, *π*). In this way, the observation sequence generated based on the proposed model can be expressed as *O*=*o*_1_*o*_2_ … *o*_*T*_, in which *o*_*t*_ stands for the vector that can be observed at the moment *t*, and *T* stands for the total observation length.

With regard to the multivariate primary nonlinear model constructed, the state transition period is a process in which the space is traversed. The sequence of spatial outputs is represented by *k*, which stands for the spatial sum that meets the similarity threshold. Thus, at the intermediate state *s*_*i*_ of this model obtained, the distribution of the corresponding observations in the class *c*^*k*^ can be expressed as the following:

(5) $$\begin{array}{c} b_{c_{k}}^{i}\left(w_{c_{i}}\right)=p\left\{k|s_{i}=w_{c_{i}}\right\}. \end{array}$$

Taking into full consideration that the distribution of *b*_*c*_*k*__^*i*^ and the spatial frequency is subject to the constraints throughout the treatment process, the greater the spatial distance, the lower the clustering level of various financial developments.

(6) $$\begin{array}{c} b_{c_{k}}^{i}\left(w_{c_{i}}\right)=\text{IFIDF}\left(i\right)=\frac{D_{c}k\left(i\right)+1}{\sum_{c}kD_{c}k\left(i\right)+|C}\times \frac{N_{c}k\left(i\right)+1}{\sum_{c}kN_{c}k\left(i\right)+|C}, \end{array}$$

where *D*_*c*_^*k*^(*i*) stands for the financial development business items that contain *w*_*c*_*i*__ in *c*_*k*_; *N*_*c*_^*k*^(*i*) stands for the number of occurrences of the space *w*_*c*_*i*__ in the class*c*_*k*_, then for the number of occurrences in the same class should have a regularization effect. The relative affiliation of the matrix to the model is denoted by *U* as the following:

(7) $$\begin{array}{c} U=\left\{u_{ik}\right\},\;\left(i=1,2,\ldots ,c;k=1,2,\ldots ,n\right), \end{array}$$

where *u*_*ik*_ stands for the affiliation of sample point *k* to the class *i* to which it falls into, which complies with the following conditions.

(8) $$\begin{array}{c} \left\{\begin{array}{cc} \sum_{i=1}^{c}u_{ik}=1, & \forall k,\\ 0\leq u_{ik}\leq 1, & \forall k,i. \end{array}\right. \end{array}$$

The aggregation center of the class *i* can be denoted by *g*_*i*_, which is

(9) $$\begin{array}{c} g_{i}=\left(g_{i1},g_{i2},\ldots ,g_{ip}\right),g_{ij}-\left[\alpha_{ij},\beta_{ij}\right],\;1\leq i\leq c,1\leq j\leq p. \end{array}$$

In the above equation, the weight of the clusters is expressed by importing the adaptive parameter *λ* as the following:

(10) $$\begin{array}{c} \lambda_{k}^{m}=\left(\lambda_{k1}^{m},\lambda_{k2}^{m},\ldots ,\lambda_{kp}^{m}\right). \end{array}$$

The combined weights can be expressed by the following equation:

(11) $$\begin{array}{c} W=\sum_{i=1}^{c}\sum_{i=1}^{n}{\left(u_{ik}\right)}^{2}\Phi \left(x_{k},g_{i}\right)=\sum_{i=1}^{c}\sum_{i=1}^{n}{\left(u_{ik}\right)}^{2}\sum_{j=1}^{p}\left[\lambda_{k}^{m}{\left(\frac{a_{kj}+b_{kj}}{2}-\frac{\alpha_{kj}+\beta_{kj}}{2}\right)}^{2}\right]. \end{array}$$

In the equation, the following conditions are met:

(12) $$\begin{array}{c} \left\{\begin{array}{c} \lambda_{ij}^{m}\geq 0,\\ \prod_{j=1}^{p}\lambda_{ij}^{m}=1. \end{array}\right. \end{array}$$

## 3. Nonlinear Empirical Analysis of the Influencing Factors of Carbon Emissions in Various Countries

This article argues that the impact of economic level growth on carbon dioxide emissions is a nonlinear relationship, mainly because the growth of economic GDP in Asian countries varies across regions, and the impact on carbon dioxide emissions is also different. Another is that because economic growth is still at different levels, this will have different effects, so it is important to determine the economic tipping point for the impact of carbon dioxide.

The sample group {*y*_*i*_, *x*_*i*_, *q*_*i*_}_*i*=1_^*n*^ is selected in this article and calculated as follows:

(13) $$\begin{array}{c} y_{i}=\theta_{1}^{\prime }x_{i}+e_{i},\;q_{i}\leq \kappa ,\\ y_{i}=\theta_{2}^{\prime }x_{i}+e_{i},\;q_{i}>\kappa , \end{array}$$

where *q*_*i*_ represents the threshold variable, *κ* represents the threshold value, and the constructed linear model *y*_*i*_=*θ*_1_′*x*_*i*_+*e*_*i*_ can be divided into two different zones, namely high and low. It should be noted that the threshold variable *q*_*i*_ can not only be used as an explanatory variable, but can also be used as an exogenous variable related to the model economy.

The nonlinear impact analysis of financial risk on carbon dioxide emissions constitutes a finite-parameter linear model. Based on satisfying the finite-parameter linear model, the finite-parameter linear model can be used for optimization according to the steady-state ecological environment of the system. In the process of dynamic monitoring of the ecological environment, the nonlinear impact of financial risks on carbon dioxide emissions can be analyzed.

A model with the following construction is called an autoregressive moving average model, simply denoted by ARMA [15]:

(14) $$\begin{array}{c} \left.\begin{array}{c} x_{t}=\phi_{0}+\phi_{1}x_{t-1}+\cdots +\phi_{p}x_{t-p}+\varepsilon_{t}-\varphi_{q}\varepsilon_{t-q}\\ \phi \neq 0,\varphi_{q}\neq 0\\ E\left(\varepsilon_{t}\right)=0,\text{Var}\left(\varepsilon_{t}\right)=\sigma_{s}^{2},E\left(\varepsilon_{t}\varepsilon_{s}\right)=0,s\neq t\\ E\left(x_{s}\varepsilon_{t}\right)=0,\forall x<t \end{array}\right\}, \end{array}$$

where *p*, *q* is called the model order, *β*=(*ϕ*_0_, *ϕ*_1_,…, *ϕ*_*p*_, *φ*_1_,…, *φ*_*q*_) ∈ *R*^*p*+*q*+1^ where (*pq*)GR_*p*_ _+_ _*q*+1_ is the model parameter. If *ϕ*_0_=0, the model is called a centralized ARMA (*p*, *q*); if *p*=0, the model is a moving average model MA(*q*). In the case of *q* = 0, the model is the autoregressive model AR(*p*).

The autocorrelation function ACF and the polarization autocorrelation function TACF are obtained by calculation, and the order of the model and the model parameter *β* can be determined [16]. The monitoring equations are as follows:

(15) $$\begin{array}{c} G_{0}=1,G_{i}=\sum_{k=1}^{i}\left(\phi_{k}^{\prime }G_{i-k}-\theta_{k}^{\prime }\right)\left(k\geq 1\right),\\ {\overset{⌢}{x}}_{t}\left(l\right)=\left\{\begin{array}{cc} \mu +\sum_{i=1}^{p}\phi_{i}{\overset{⌢}{x}}_{t}\left(l-i\right)-\sum_{i=l}^{q}\phi_{i}\varepsilon \left(t+l-i\right), & l\leq q,\\ \mu +\sum_{i=1}^{p}\phi_{i}{\overset{⌢}{x}}_{t}\left(l-i\right), & l>q, \end{array}\right.\\ \text{Var}\left(e_{t}\left(l\right)\right)=\sum_{i=0}^{l-1}G_{i}^{2}\sigma_{\varepsilon }^{2},\;\forall l\geq 1, \end{array}$$

where

(16) $$\begin{array}{c} \phi_{k}^{\prime }=\left\{\begin{array}{cc} \phi_{k}, & 1\leq k\leq p,\\ 0, & k>p. \end{array}\right.\\ \phi_{k}^{\prime }=\left\{\begin{array}{cc} \theta_{k}, & 1\leq k\leq q,\\ 0, & k>q. \end{array}\right.\\ {\overset{⌢}{x}}_{t}\left(k\right)=\left\{\begin{array}{cc} {\overset{⌢}{x}}_{t}\left(k\right), & k\geq 1,\\ x_{t+k}, & k\leq 0. \end{array}\right. \end{array}$$

*σ*_*ε*_^2^ can be replaced by the sample variance *σ*_*ε*_^2^: where *e*_*i*_ is the error between the alarm value and the actual observed value using the 1-step alarm equation.

(17) $$\begin{array}{c} {\hat{\sigma }}_{\varepsilon }^{2}=\left(\frac{\sum_{i=1}^{t}{\left(e_{i}-\bar{e}\right)}^{2}}{\left(t-1\right)}\right),\bar{e}=\sum_{i=1}^{t}\left(\frac{e_{i}}{t}\right). \end{array}$$

*P*(*t*) is the monitoring value at time *t* obtained by the PIE remote monitoring image processing algorithm. Let $\varepsilon =\lambda \sqrt{\left(1+\varphi_{1}^{2}+\cdots +\varphi_{q}^{2}\right)\sigma_{\varepsilon }^{2}}$, *λ* > 1, be a constant, and the interval does not contain the real value at time *t* with the highest probability. According to the input *λ* value, the monitoring interval corresponding to the probability can be obtained, and the above algorithm is implemented in the system to achieve the purpose of warning monitoring data.

Ecological environment detection and real-time risk monitoring are of great significance for ecological environment-related resource distribution, flow planning service level, and safety monitoring [17, 18]. According to the obtained data, it is used to analyze the ecological environment performance, analyze the ecological environment operation state and diagnose the cause of the failure, and can also be used to monitor the cause of the failure. Ecological environment monitoring and real-time risk alerts are important manifestations of ecological environment management and systematic integration, providing detailed data information for the operation and maintenance of the ecological environment. It plays an important role in ecological environment performance analysis, abnormal monitoring, link status monitoring, and capacity planning. As the focus of current research in this field, ecological environment monitoring can be perfectly combined with different industries to complete the full use of data from different industries in the actual ecological environment monitoring environment.

With regard to the analysis of the nonlinear effect of financial risks on carbon dioxide emissions, a finite-parameter linear model is established, which can be used based on complying with the finite-parameter linear model. In accordance with the steady-state ecological environment of the system, the optimal solution can be obtained. During the process of monitoring the dynamic changes in the ecological environment, financial risks can be used to analyze the nonlinear influence on carbon dioxide emissions. With regard to the issues analyzed above, the green investment demand function is used in this article, which is expressed as follows:

(18) $$\begin{array}{c} w=\alpha L_{Y}^{\alpha -1}\int_{0}^{A}x{\left(i\right)}^{1-\alpha }\text{d}i,\\ p\left(i\right)=\left(1-\alpha \right)L_{Y}^{\alpha }x{\left(i\right)}^{-\alpha }. \end{array}$$

Ecological environmental protection is the foundation for the construction of ecological civilization construction, and the implementation of real-time, rational, and accurate monitoring of ecological environmental protection can also provide a theoretical basis for analyzing the decisions made by the relevant authorities of environmental protection and inspection. With regard to a large number of emerging economic and ecological transformation projects that have been emerging constantly, it is of important significance to analyze the issues and defects in the process of ecological environmental protection in detail so as to develop effective training programs and improvement plans in the later stage. In the process of analyzing the evolution of ecolocal environment protection during the ecological transformation of traditional emerging economies, ecological environment protection and real-time risk alerts are also effective processes for data acquisition and analysis to achieve the goal of protecting the ecological environment. The index data are collected from the ecological environment, and the corresponding feedback is given. The data obtained are used to analyze the performance of the ecological environment, diagnose the root cause of faults, and monitor the root cause of the related faults.

The analysis of the financial risk factor is mainly carried out by collecting all analysis data on the nonlinear effect of carbon dioxide emissions, which are saved in a data storage device with a high capacity. After the application of data screening, processing, and cleansing technologies and the relevant information, they are transferred to the corresponding applications to perform the procedures and collect data on the platform regarding the features of public use of nonlinear impact analysis data of carbon dioxide emissions quickly and accurately.

(19) $$\begin{array}{c} T\left(a,a_{1}\right)=\frac{\sum_{i=1}^{n}\left({\left(q_{i}-s\right)}^{2}\left(q_{i}-s-l\right)\right)\left(q_{i}-s^{2}\left(q_{i}-s-l\right)\right)}{\sqrt{\sum_{i=1}^{n}{\left(q_{i}-s^{2}{\left(q_{i}-s-l\right)}^{2}\right)}^{2}+{\left(q_{i}-s^{2}{\left(q_{i}-s-l\right)}^{2}\right)}^{2}}}, \end{array}$$

where *T*(*a*, *a*_1_) stands for the set of characteristic attributes of carbon dioxide emission nonlinear effect analysis by using the relevant data and the carbon dioxide emissions used for the characteristic expressions in the nonlinear effect analysis; *q*_*i*_ stands for the number of data features after the classification of data on the carbon dioxide emissions used for the nonlinear impact analysis; *s* stands for the characteristic content of the nonlinear impact analysis of carbon dioxide emissions. As a numerical parameter, it is a feature specific to the carbon dioxide emission nonlinear effect analysis. After the features of the data used for the nonlinear impact analysis of carbon dioxide emissions are identified, the non-characteristic attributes should be removed, and the equation for the removal of the redundant data is shown as the following:

(20) $$\begin{array}{c} L=\overset{⟶}{q}+\frac{\sum_{i=1}^{n}{\left(T\left(a,a_{1}\right)\right)}_{i}\left(q-e\right)}{\sum_{i=1}^{n}{\left[T\left(a,a_{1}\right)\right]}_{i}^{2}}, \end{array}$$

where *L* is used to define the removal benchmark and remove those that fail to comply with the benchmark. $\overset{⟶}{q}$ stands for the filtering request used for removal; *e* stands for the existing redundant data removal request. Thus, the features of the data can be obtained by filtering. In the aspect of adjustment in the economic scale, it can attract a large amount of private and social capital to enter the green economy market, which will expand the financing channels in Asian countries, increase the cash holdings of Asian countries, and address the issues of the insufficient green economy in Asian countries, especially in the Asian countries with environmental protection initiatives based on technology. In accordance with the results of the study, the relationship between the growth of emerging economies and environmental sustainability can be observed [19]. In the case of the increasing GDP per capita in various countries, the degree of environmental sustainability also presents a trend of first decreasing, then increasing, and finally declining. The economic analysis model established for each country allows for an in-depth analysis and evaluation of the relevant economic development factors and the assessment of the factors affecting the development of the economy in each country and the environmental sustainability of the factors influencing the growth of their economy. In this way, the accuracy of analyzing the sustainability of the green economy can be improved quickly, which can also promote the effective utilization of economic resources. In a green economy environment, the rapid restructuring of the economy in each country can play a complementary role in environmental protection.

As an emerging Asian economy with a relatively high degree of economic development and openness, the emergence of domestic trade and investment protectionism will lead to slow economic and trade development and will seriously affect financial difficulties. According to the continuous development of various factors such as big data, artificial intelligence, and blockchain, more traditional industries will begin to change continuously. At present, with the development of financial technology, different types of electronic payment models have begun to develop on a large scale. The continuous development of traditional financial enterprises will accelerate the “disintermediation,” and the cross-border flow of funds within countries will become faster and more convenient.

## 4. Analysis of Examples and Results

In this article, the minimum value of Cronbach's *α* corresponding to the relevant solved is 0.881 (Table 1). At the same time, it is necessary to remove any question item; otherwise, the Cronbach's *α* obtained will not be significantly improved. The minimum value of the factor loading calculated is 0.644, the value obtained for KMO is greater than 0.7, and the minimum value of the cumulative variance contribution obtained through the operation is 55.40%. From the above results, it can be concluded that the reliability of the experimental data is relatively high. In the scale validity tests of CR and emissions, all the values for the variable CR obtained are 0.8 or so, and the values of emissions are no less than 0.5 on average. Hence, it can be concluded that the convergent validity of the experimental process is relatively high as well. The square root of all the values of the variable emissions is greater than the magnitude of the correlation coefficient of the two variables, which suggests that the discriminant validity of the samples obtained is relatively high.

With regard to the phenomenon of the reduced validity of the model training results, to reduce the unbalanced data set effectively, a method of deficiency sampling for multiple classes and oversampling for a few classes is adopted in this experiment to generate a relatively balanced data set. The analysis results of the training data set with 300,000 pieces of data collected indicate that the ratio of majority and minority classes after sampling is 9 : 1 to 11 : 003 that of the raw data, which indicates that the unbalanced feature of the data set has been effectively improved. Table 1 below shows the comparison in the performance of the data set after sampling and the data set without sampling.

The established model is adjusted for a number of times and validated against the data in the data set. The overdue rates without using the model and with using the model are compared (Figure 1).

For the threshold likelihood ratio test that can represent the level of economic development in the region, the test results are shown in Figure 1. Figure 1 shows the likelihood ratio verification at the second threshold ln*Y*. According to the test results in Figure 1, it can be seen that without considering that the likelihood ratio corresponding to the second threshold estimated value is 0. In order to avoid the existence of other estimated values below the threshold in the entire area, it can be determined that the third threshold does not exist.

In this article, the influence of financial risks on carbon dioxide emissions is explored through data analysis by establishing a model based on financial risks and carbon dioxide emissions. The effects of financial risks on the limits of carbon dioxide emissions in different dimensions can hardly be determined, and there is a certain similarity in the relationship between financial risks and carbon dioxide emission limits. In the green investment and fierce economic competition with respect to the huge amount of inputs against the financial risks, it has substantially reduced the emissions of carbon dioxide compared with the traditional policies and regulations. Thus, it has a positive influence in boosting the long-term growth of the domestic economy; it can not only speed up the economic growth effectively but also achieve the optimization of the economic structure of the green investment. As the financial risks can play a certain role in limiting the emissions of carbon dioxide, it is also necessary to develop the proportion of green economy investment vigorously, which will also have a certain influence on the ecological innovation.

Under different policies for environmental protection, the level of the effect that financial risks have on carbon dioxide emissions is also decreasing constantly. Thus, in the nonlinear effect analysis, carbon dioxide emissions show an interaction with the financial risks. In accordance with the test results, it can be known that for Asian countries, in the process of nonlinear effect analysis of carbon dioxide emissions, the probability outlier that mainly reflects the financial risk process is also relatively low. In Figure 2, the horizontal axis indicates the level of analysis on the nonlinear effect of carbon dioxide emissions, and the vertical axis indicates that there can be a difference in the probability of engaging in entrepreneurial activities with financial risks and without financial risks. It is assumed that the upper and lower bounds of the 85% confidence interval are above or below the 0 horizontal line. With the gradual increase in the nonlinear effect of carbon dioxide emissions, the impact of financial risks on the carbon dioxide emissions starts to decline. If the carbon dioxide emissions obtained are less than 74.97, the impact of financial risks on the carbon dioxide emissions will only present a positive and significant relationship; if it exceeds the threshold value, the impact of financial risks on the carbon dioxide emissions will not be significant.

In this article, the limitation effect of carbon dioxide emissions is tested, and the test results are shown in Table 2. It can be concluded from the table that the financial risks have a positive effect on the carbon dioxide emissions (*β* = 0.615, *p* < 0.01). At the same time, the green economy also has a significant positive effect on the analysis of the nonlinear effect of carbon dioxide emissions. However, the regression coefficient of the effect of financial risks on the analysis of the nonlinear influence of carbon dioxide emissions will be reduced from 0.615 to 0.337. Thus, the green economy plays a partial mediating role in the relationship between the financial risks and the carbon dioxide emissions in the nonlinear impact analysis.

To achieve sustainable development with environmental protection in the national economies of Asian countries, it is necessary to make effective use of the nonlinear effect analysis of carbon dioxide emissions under the financial risks of the system. As a new driver for the green economy, financial risks are analyzed from the perspective of coordinated development of the economy and environmental protection. In this article, the mutual impacts of the green economy on financial risks are thoroughly analyzed. Based on the presence of the intrinsic links, financial risks in the nonlinear effect analysis of carbon dioxide emissions is conducive to driving the economic growth, while playing a continuous role in the improvement of the environment. The proportion of resource consumption is also relatively high in regions with a high level of economic growth. Driven by the financial risk factors, it can effectively reduce environmental pollution in the green economy and further boost the economic growth and reduce the carbon dioxide emissions. The results of the practical case analysis indicate that: In the proportion of heavy investment in the green economy, environmental sustainability has been greatly improved as compared to the traditional economic development model. This has a positive effect on driving the long-term economic growth of Asian countries, which can not only accelerate the economic growth effectively but also achieve the optimization of the economic structure in the Asian countries.

In this article, the root test (ADF) is used to test different variables. The test results are shown in Table 3, where *c*, e, *y*, *y*2, d*y*, and *o* are expressed as level and trend nonstationary time series in turn, but all variables are first order. There is a causal relationship between financial risk and environmental quality. Therefore, to use the constructed model to evaluate, it is necessary to use the Granger causality test to test the relationship between carbon dioxide emissions and the growth of economic development. According to the test results in Tables 4 and 5, it can be seen that there is a significant causal relationship between the above two variables.

According to the test results, there is a negative correlation between financial risks and carbon dioxide emissions in Asian countries. From the specific details, the evaluation coefficient of 0.35 means that the growth rate of financial risks in this region will reduce carbon dioxide emissions from 1% to 0.35%. There is an obvious positive correlation between energy consumption and carbon dioxide emissions. The sign of the detected regression coefficient is similar to the theoretical value, and the coefficient value is 0.31, indicating that the per capita energy consumption in the region increases by 1%. From a long-term perspective, carbon dioxide emissions can be increased to 0.31%, and the level coefficient of per capita GDP at the level of 5% is also 3.2, indicating that for every 1% increase in per capita income, carbon dioxide emissions will rise to 3.2%.

## 5. Conclusion

Based on the regional differences in carbon emissions and GDP economic development in the current Asian environment, this article proposes measures on the factors affecting carbon emissions from economic growth and estimates and tests based on the revised STIRPAT module. By studying the situation of CO_2_ emissions in economically developing regions, the findings are shown to be nonlinear. Under the environment of a low level of economic development in GDP, there is a direct relationship between the faster economic development and carbon emissions. Asia has expressed its commitment to climate development, forced the development of low-carbon life, and made real improvements through carbon reduction. This improvement determines the change of quality of the living environment and shoulders the burden of social responsibility. At the same time, it is a long development process to rectify and develop the structure of the industry. In the implementation stage, the emission reduction needs to be maximized. The Asian environment under study has entered a new course. The differences in the economic development and economic situation of each place have a decisive effect on the local carbon emissions. It requires lower carbon, greener, and less energy consumption to generate the largest GDP economy benefit.

## Figures and Tables

**Figure 1:** Comparison of the overdue rate without using the model and with using the model.

**Figure 2:** Impact of financial risks on carbon dioxide emissions.

**Table 1:** Comparison of sampling effects of the experimental samples.

Training set	Test data set			Validation data set		
	Accuracy rate (%)	Recall rate (%)	F1 value (%)	Accuracy rate (%)	Recall rate (%)	F1 value (%)
Without sampling	35.82	41.01	38.20	31.01	35.24	33.09
Comprehensive sampling	52.58	67.47	59.11	36.86	39.77	38.26

**Table 2:** Results of nonlinear impact analysis of the relationship between financial risks and carbon dioxide emissions.

Variables	Green economy		Analysis of the nonlinear effect of carbon dioxide emissions			
	Parameter 1	Parameter 2	Parameter 1	Parameter 2	Parameter 3	Parameter 4
Scale of national economy	−0.018	−0.03	0.094	0.09	0.104	0.098
Type of national economy	−0.04	0.01	−0.075	−0.01	−0.053	−0.08
Financial risks		0.615^*∗∗*^		0.551^*∗∗*^		0.337^*∗∗*^
Green economy					0.553^*∗∗*^	0.347^*∗∗*^

**Table 3:** ADF check result.

	ADF	*K*
*c*	−1.23	1
*e*	0.93	0
*y*	0.92	1
*y*2	1.33	1
d*y*	1.52	1
*o*	−1.52	0
Δ*c*	−4.34	1
Δ*e*	−3.11	0
Δ*y*	−3.23	0
Δ*y*2	−4.11	1
Δd*y*	−4.03	1
Δ*o*	−4.23	0

**Table 4:** Granger causality test results.

Null hypothesis	*F*-statistics	Prob.
*c* does not Granger cause *y*	0.42	0.63
*y* does not Granger cause *c*	3.16	0.02

**Table 5:** ADRL estimation results.

	Model 1	Model 2	Model 3	Model 4
Cointegrating check				
*F*-statistics	6.74	5.81	07.94	6.81
ARDL estimation				
Intercept	−7.6^*∗∗∗*^ (−2.6)	−6.2^*∗*^0 (−1.8)	−4.23^*∗∗*^ (−11.64)	−5.91^*∗∗∗*^ (−2.38)
e	00.31^*∗∗∗*^ (0.21)	000.68^*∗∗∗*^ (3.46)	NA NA	NA NA
*y*	3.21^*∗*^ (1.73)	3.53^*∗∗∗*^ (2.47)	3.15^*∗∗*^ (1.89)	2.86^*∗∗∗*^ (2.34)
*y*2	NA NA	−0.53^*∗∗∗*^ (−2.42)	NA NA	−0.45^*∗∗*^ (−2.14)
d*y*	−0.35^*∗∗∗*^ (−2.89)	−0.27^*∗∗*^ (−2.18)	−0.67^*∗∗∗*^ (−2.38)	−0.17^*∗∗∗*^ (−1.98)
tr	0.56^*∗∗*^ (2.00)	0.23^*∗∗∗*^ (2.98)	0.19^*∗*^ (1.67)	0.89^*∗∗∗*^ (4.72)

*Note.* ^*∗∗∗*^ means significant at 1% level, ^*∗∗*^means significant at 5% level, ^*∗*^ means significant at 10% level.

## Data Availability

The data that support the findings of this study are available from the corresponding author upon request.
